The article "Clinical Effect of the Guizhi Shaoyao Zhimu Decoction in the Treatment of Hyperuricemia" was retracted in 2024. Reasons: signs of a paper mill; suspected computer-generated content; unreliable results or conclusions; concerns about the data.

# Clinical Effect of the Guizhi Shaoyao Zhimu Decoction in the Treatment of Hyperuricemia

**DOI:** 10.1155/2022/5186210

**Published:** 2022-08-24

**Authors:** Qilin Yang, Jikong Zhang, Jiuwei Li

**Affiliations:** ^1^Hongxingtang Pharmacy, Shizhong District, Zaozhuang, Shandong 277100, China; ^2^Information Center, The Second Affiliated Hospital of Shandong University of Traditional Chinese Medicine, Jinan, 250000 Shandong, China; ^3^Medical College of the Second Clinical College, Shandong University of Traditional Chinese Medicine, Jinan, 250000 Shandong, China

## Abstract

Traditional Chinese Medicine (TCM) is a medical system with a distinctive theoretical framework and extensive experience in identification and treatment acquired by the Chinese people in long-term medical practice and life practice. It is a complete, integrated, and complex knowledge system in epistemology. This study is aimed at exploring the clinical effectiveness of TCM called the Guizhi Shaoyao Zhimu Decoction in the treatment of hyperuricemia. A total of 100 patients with hyperuricemia at the Medical College of the Second Clinical College, Shandong, China, from January 2019 to January 2022 are selected as the research subjects and divided into group A and group B according to the random table method, with 50 cases in each group. Group A is treated with oral allopurinol tablets, 100 mg, 2 times a day, and group B is treated with the modified Guizhi Shaoyao Zhimu Decoction based on group A. For observation, serum uric acid (SUA) levels, urinary uric acid (UUA) levels, levels of serum inflammatory response factors (IL-6, CRP, and TNF-*α*), vascular endothelial function indexes (serum malondialdehyde (MDA) content, nitric oxide (NO) content), an acute attack of gout, and the incidence of adverse reactions are measured. Results show that after 2 w and 4 w of treatment, the levels of blood uric acid in each group gradually decreased compared with those before treatment, and group B is lower than group A (*P* < 0.05). After treatment, the vascular endothelial function indexes and inflammatory factor levels in each group are significantly improved compared with those before treatment, and the indexes in group B are better than those in group A. There is no significant difference in the incidence of related adverse reactions and acute attack of gout (*P* > 0.05). This shows that the TCM Guizhi Shaoyao Zhimu Decoction has a significant curative effect in the treatment of patients with hyperuricemia, which is worthy of clinical reference application.

## 1. Introduction

Hyperuricemia (HUA) is a metabolic disorder caused by increased uric acid levels and/or reduced uric acid excretion. HUA is often defined as fasting serum uric acid levels > 420 *μ*mol/L in men and menopausal women or >357 *μ*mol/L in premenopausal women on two different days under a normal chow diet [1]. Its clinical characteristics include recurrent gouty acute arthritis caused by HUA, tophi deposition, tophi-induced chronic arthritis, joint sclerosis, chronic interstitial inflammation, uric acid nephrolithiasis, and the formation of gouty nephropathy [2].

The article "Clinical Effect of the Guizhi Shaoyao Zhimu Decoction in the Treatment of Hyperuricemia" was retracted in 2024. Reasons: signs of a paper mill; suspected computer-generated content; unreliable results or conclusions; concerns about the data.

The incidence of HUA in developed countries is 5%. Epidemiological studies show that the prevalence of HUA and gout has recently been increasing globally [3]. According to population-based studies, the prevalence of HUA in Western populations is believed to be around 21%, and that of gout is between 1% and 4% [4]. Based on the survey of National Health and Nutrition Examination (2007–2016), a prevalence of 20.1% and 20.3% for HUA was reported among men and women, respectively, in America from 2015 to 2016 and the occurrence of HUA remained constant from 2007 to 2016 [5, 6]. In China, rapid economic growth has caused dietary changes, especially an increase in the intake of high-purine diets, which has increased the incidence of HUA. A meta-analysis performed in 2011 revealed that 8.5% of women and 21.7% of males in China have HUA. The several potential side effects of HUA could significantly raise the cost of healthcare. Therefore, it is crucial to consider HUA in China and worldwide [7].

HUA is asymptomatic, and its onset is insidious, so it is often ignored by patients, but it causes great harm [8]. And for a long time, HUA has not received enough attention because it is considered to be a simple metabolic disease, but since the late 1980s, more and more studies have found that HUA is not only a cause of gouty arthritis and kidney stones. The pathological basis of renal failure and high uric acid can cause damage to multiple systems and is closely related to metabolic syndrome diseases such as hypertension, atherosclerosis, heart disease, blood lipid and blood glucose metabolism disorders, obesity, and insulin resistance [9]. Therefore, how to prevent and treat HUA safely and effectively has become an important topic of increasing concern in the medical community.

The basic research on hyperuricemia in modern medicine has made great progress, but the clinical treatment of HUA is not ideal [10]. TCM has made great progress in the treatment of HUA. TCM has the advantages of being safe and effective, can effectively improve clinical symptoms, and has gradually attracted attention [11]. It is believed that the effectiveness of the primary components of TCM extracts in treating HUA is due to their active components. Colchicine is present in the Pseudobulbus Cremastrae seu Pleiones bulbs, which are employed in decoctions by Zhang et al. [12] and Li [13] and others. Additionally, the glabrous greenbrier rhizome, which has astilbin as an active component, is present in the Chinese medicinal herbs utilized by Zhou [14], Yu [15], Tan et al. [16], and Li [13]. Several herbs have also been used, including the seven-lobed yam rhizome [17], Job's tear seeds [18], and Radix Achyranthis Bidentatae [19], all of which improve different physiological processes, such as uric acid excretion promotion, platelet accumulation reduction resulting in improved microcirculation, and anticoagulant function. The Guizhi Shaoyao Zhimu Decoction (GSZD) is a representative formula of Zhongjing for treating dampness and chronic disease. Clinical pharmacological studies have shown that it can reduce gouty joints. It can prevent the creation of inflammatory pain factors, inhibit inflammatory mediators such as prostaglandins, leukotrienes, IL-6, and TNF-*α*, induce apoptosis, regulate T cell function, and inhibit osteoclast activation [14, 15]. Therefore, this study mainly observed the clinical effectiveness of GSZD in the treatment of HUA and provided some references for the clinical treatment of HUA. From January 2019 to January 2022, a total of 100 patients with HUA at the Second Clinical College of Shandong, China, were selected as the study participants. Using the random table approach, 50 cases from each group were separated into groups A and B. Oral allopurinol tablets, 100 mg, were given to group A twice a day, and group B was treated with GSZD. Results revealed that the blood uric acid levels gradually declined throughout treatment in both groups and that the uric acid level of all individuals in group B was lower than that of group A's individuals after two weeks and four weeks.

The article "Clinical Effect of the Guizhi Shaoyao Zhimu Decoction in the Treatment of Hyperuricemia" was retracted in 2024. Reasons: signs of a paper mill; suspected computer-generated content; unreliable results or conclusions; concerns about the data.

The remaining manuscript is organized into the following sections.  Section 2 provides a detailed description of the study subjects and treatment method. The results are presented in Section 3. The results are analyzed in Section 4, and Section 5 is about the conclusion.

## 2. Methods

### 2.1. Subjects

A total of 100 patients with hyperuricemia from the Medical College of the Second Clinical College, Shandong, China, from January 2019 to 2022 were selected as the study subjects. They were divided into group A and group B according to the randomization method (coin toss method), with each group having 50 patients. Group A had 27 males and 23 females, aged 46-56 years (mean51.18 ± 2.54years), and group B included 28 males and 22 females, aged 46-55 years (mean50.72 ± 2.07years). The general information of both groups was the same (*P* > 0.05), which could be compared. The diagnostic criteria included fasting serum uric acid content of >420 *μ*mol/L in men and menopausal women or >357 *μ*mol/L in premenopausal women [20–22].

The inclusion criteria were as follows: (i) the patients who did not participate in other clinical investigators within 1 month of enrollment, (ii) those who were not allergic to and tolerated the drugs used in this study, (iii) all women who were postmenopausal, and (iv) family members and patients. All who signed written information consent voluntarily participated in the study.

The exclusion criteria were as follows: (i) all patients with secondary HUA, such as myeloma, leukemia, polycystic kidney disease, renal failure, and certain endocrine diseases, including certain drugs, such as aspirin, diuretics, and antituberculosis drugs, as well as uric acid; (ii) those with mental illness who cannot communicate; (iii) women who are pregnant or breastfeeding; (iv) those with other vital organ dysfunctions; and (v) those who had received other treatments before participating in the study.

### 2.2. Methods

Both groups of patients received routine health education, and they were instructed to adjust their lifestyle and dietary structure, including avoiding a high-purine diet; for obese patients, it is recommended to adopt a low-calorie balanced diet and increase exercise to avoid obesity. Maintain ideal body weight and quit drinking all kinds of alcohol, especially beer. Similarly, daily water intake should be more than 2000 mL to maintain urine output. Patients in group A were added with allopurinol (Guangzhou Baiyunshan Pharmaceutical Group Co., Ltd., H44021492), 100 mg, orally, twice a day, and maintained at 100-200 mg after serum uric acid was normal. For group B based on group A (Shangyu Guizhi Shaoyao Zhimu Decoction), the formula is composed of Guizhi 12 g, Mahuang 6 g, Baishao 12 g, Anemarrhena 9 g, Fangfeng 9 g, Duhuo 12 g, Atractylodes 9 g, Asarum 3 g, Heifu tablet 10 g (decorated first), Tripterygium wilfordii 9 g (fried first), and licorice 6 g. For those with cold, dry ginger 6 g, epimedium 15 g, and cinnamon 6 g were used; for heat evil, 9 g phenol, 9 g phellodendron, 12 g honeysuckle, and 9 g fried gardenia were used. For those with anorexia, 15 g of chicken Neijin, 9 g of perilla stem, and 9 g of Jiao Sanxian each were used. In the case of an acute attack, Heifu Pian, Guizhi, Codonopsis, Jiawei Lingxian 15 g, plantain seed 20 g (fried in cloth), Shiwei 15 g, Corydalis 15 g, Tuckahoe 30 g, and honeysuckle vine 20 g were used; 1 dose/d was followed. Both groups were treated for 4 weeks.

### 2.3. Observation Indicators

Serum uric acid (SUA) levels and 24 h urinary uric acid (UUA) excretion were detected before treatment and at 2 weeks and 4 weeks after treatment. Next, the fasting blood samples were acquired from patients before and after treatment and centrifuged to get the supernatant; the ELISA method (Abcam, ab178013) [23] was used to measure the level of interleukin-6 (IL-6), and the ELISA method (Abcam, ab181421) [24] was employed to measure the tumor necrosis factor-*α* (TNF-*α*) level. Likewise, the ELISA method (Abcam, ab260058) [25] was used to measure the C-reactive protein (CRP) level [26]. Moreover, from all the patients, fasting blood was obtained before and after treatment, and serum malondialdehyde (MDA) [19] content was detected by the thiobarbituric acid method, and nitric oxide (NO) [27, 28] content was detected by the nitrate reductase method. The occurrence of adverse reactions and the acute attack of gout during treatment were recorded in the two groups.

The article "Clinical Effect of the Guizhi Shaoyao Zhimu Decoction in the Treatment of Hyperuricemia" was retracted in 2024. Reasons: signs of a paper mill; suspected computer-generated content; unreliable results or conclusions; concerns about the data.

### 2.4. Analysis

The SPSS V27.0 [29–31] statistical software was employed for statistical analysis and measurement. The data were expressed as mean ± standard deviation ($\bar{x}\pm s$) (*n*, %), and a *t*-test was used for statistical analysis. The *P* < 0.05 specified a statistically significant difference between the two groups.

## 3. Results

### 3.1. Comparison of Blood Uric Acid Levels at Different Observation Points

Before treatment, there was no change between the two groups in terms of the blood uric acid levels of any of the patients in groups A or B (*P* > 0.05). After two and four weeks of treatment, the blood uric acid level in the blood of each group slowly declined as compared with the uric acid level before treatment. Similarly, the uric acid level of individuals in group B was lower significantly lower than that in group A (*P* < 0.05).  Table 1 provides the comparative results for uric acid levels in both groups before and after treatment.

### 3.2. Comparison of Vascular Endothelial Function Indexes

Table 2 provides a comparison of the vascular endothelial function indexes before and after treatment for both groups. Before treatment, the serum MDA and NO levels in all patients were the same (*P* > 0.05). After treatment, the vascular endothelial function indexes in each group were measured and found to be significantly improved compared with those before treatment. The vascular endothelial function indexes in group B were better than those in group A (*P* < 0.05).

### 3.3. Comparison of Inflammatory Factor Levels

Table 3 shows that there was no significant difference in the levels of serum TNF-*α*, IL-6, and CRP in each group before treatment (*P* > 0.05). However, after treatment, there is a significant difference between the inflammatory factor levels of both groups A and B (*P* < 0.05).

The article "Clinical Effect of the Guizhi Shaoyao Zhimu Decoction in the Treatment of Hyperuricemia" was retracted in 2024. Reasons: signs of a paper mill; suspected computer-generated content; unreliable results or conclusions; concerns about the data.

### 3.4. Comparison of 24 h Uric Acid Levels in Each Group

The comparative results for 24-hour uric acid levels before and after treatment are given in Table 4. It is obvious that before treatment, the uric acid levels in each group are the same (*P* > 0.05). After treatment with GSZD for two weeks and four weeks, the level of uric acid in group B was higher than that before treatment, and group B was higher than group A which shows a statistically significant difference between the uric acid levels of all the individuals in both groups (*P* < 0.05).

In group A, 3 patients had different degrees of gastrointestinal discomfort, which were relieved spontaneously, and 2 patients had acute gout attacks; group B had no drug-related adverse reactions and no acute gout attack. Between the two groups, there was no apparent difference in the frequency of drug-related side effects and acute gout attacks (*P* > 0.05).

## 4. Discussion

Hyperuricemia refers to a state in which the blood uric acid concentration in the human body continues to increase, and it is a chronic metabolic disease caused by purine metabolism disorders. According to relevant reports [32, 33], HUA is currently showing a high incidence in the world, and its occurrence is closely related to the changes in the diet structure, the living habits of modern people, the acceleration of the global aging process, and the use of clinical drugs [34]. Although most people with HUA have no obvious clinical symptoms due to the long-term and gradual increase and effect of serum uric acid (SUA) in the blood, there are still some patients with gouty arthritis, uric acid nephropathy, and other diseases [35]. In addition to joint swelling, pain, and deformity in bones, in severe cases, patients may die due to chronic renal failure. A large number of domestic and foreign studies have also shown that HUA is also closely associated with the incidence and development of hyperlipidemia, diabetes, coronary atherosclerosis, cerebral infarction, tumors, and other diseases. This can also increase cardiovascular and cerebrovascular diseases, metabolic syndrome, and tumors. Therefore, early intervention and treatment of HUA have positive significance in delaying the occurrence of related complications and improving the prognosis of patients. At present, in addition to dietary control and lifestyle intervention, most patients with HUA are treated with Western oral medicines. Although the curative effect is good, some medicines have obvious adverse reactions and long-term use of patients has poor compliance to achieve the desired effect.

The article "Clinical Effect of the Guizhi Shaoyao Zhimu Decoction in the Treatment of Hyperuricemia" was retracted in 2024. Reasons: signs of a paper mill; suspected computer-generated content; unreliable results or conclusions; concerns about the data.

With the improvement of modern medicine and healthcare technology, there are more and more modern studies on the treatment of HUA with TCM. Several studies have confirmed that TCM has a good effect on improving the clinical symptoms of patients and reducing the level of blood uric acid in HUA patients [36, 37]. In terms of safety, TCM has the characteristics and advantages of naturalness and low toxicity. Through drug compatibility, processing, decoction, and other methods, the toxic and side effects of the drug itself and between drugs can be effectively reduced. The adverse reactions are small, and the patients find the drug easy to tolerate. In recent years, the combined use of Chinese and Western medicines has been widely recognized in clinical practice. In Wang et al.'s [32] animal experiments, Sanmiao pills can successfully decrease SUA levels in mice, and its mode of action may be related to the prevention of xanthine oxidase (XO) activity [38]. The earliest understanding of HUA started from the research on gout and other related complications caused by it. Because gout often has symptoms such as pain in limbs and joints, low back pain, edema, and difficulty urinating, physicians in the past dynasties often classified it as “arthralgia,” “white tiger calendar festival,” “walking note wind,” “edema,” and “stone stranguria.” The pathogenesis is mainly due to the lack of congenital endowment, exogenous pathogenic qi, improper diet, old age, and frailty. The serum uric acid level is an objective test indicator. The serum uric acid test in HUA patients is the standard for the diagnosis of HUA. The curative effect of HUA patients can be reflected by the improvement of serum uric acid levels. This study showed that the improvement of the SUA level in group B was significantly lesser than that in group A, and the level of uric acid was significantly increased in group A (*P* < 0.05), suggesting that the TCM Guizhi Shaoyao Zhimu Decoction can effectively reduce the level of SUA and promote the excretion of uric acid. The combined treatment of HUA with allopurinol is more effective than allopurinol alone.

Studies have found that “serum UA at 60-120 mg/L can upregulate the expression of CRP mRNA in vascular smooth muscle cells and umbilical vein endothelial cells, increase the release of CRP into the cell culture medium, and inhibit p38 or extracellular signal-regulated kinase 44 or regulated kinase 42.” Reduce UA-induced CRP expression [39]. CRP may be involved in the vascular remodeling effect induced by UA, and UA can change the propagation, migration, and NO release of human vascular cells by inducing the expression of CRP [29]. Activated monocytes are the main source of serum IL-6. Lymphocytes, endothelial cells, hepatocytes, and adipocytes can all produce IL-6. The main biological role of IL-6 is to regulate the immune response and hematopoietic system and induce acute phase proteins [40]. TNF-*α* is a primary cytokine in the inflammatory network chain, is an important proinflammatory mediator, and can be stimulated by uric acid. Crystallization stimulates and increases the expression of other inflammatory factors and can upregulate the expression of adhesion molecules, and they interact and influence each other to aggravate tissue damage and inflammation. This study showed that the serum levels of IL-6, CRP, and TNF-*α* in group B were significantly lower than those in group A (*P* < 0.05), which confirmed the inhibitory effect of the Guizhi Shaoyao Zhimu Decoction on inflammatory factors in the body as similar to the findings of Hui et al. [21].

The article "Clinical Effect of the Guizhi Shaoyao Zhimu Decoction in the Treatment of Hyperuricemia" was retracted in 2024. Reasons: signs of a paper mill; suspected computer-generated content; unreliable results or conclusions; concerns about the data.

This study proposes that the combination of allopurinol and GSZD in the treatment of HUA can more effectively inhibit the body's inflammatory response. Most patients with HUA have hyperlipidemia, inflammatory response, and vascular endothelial injury, and these factors may affect the development of HUA. Moreover, the vascular endothelial function indexes of patients in group B were significantly improved compared with those in group A (*P* < 0.05), suggesting that GSZD combined with a modified recipe could effectively improve the vascular endothelial function in patients with HUA. Guizhi and Mahuang have the effects of dispelling wind and drenching yang. Atractylodes and Fangfeng can dispel wind and remove dampness. Shaoyao Zhimu can nourish yin and reduce swelling. Aconite can warm meridians, disperse cold, and relieve pain. Licorice and ginger can nourish the stomach and regulate the middle. The whole formula has the effect of dispersing wind, dispelling cold and dampness, activating yang, and eliminating paralysis. In addition, the incidence of drug-related adverse reactions in group B was lower than that in group A, but the difference was not statistically significant (*P* > 0.05), which may be due to the insufficient sample size in this study. The study will expand the sample size to clarify the efficacy of the combination of allopurinol and GSZD in the treatment of HUA and provide new ideas and new solutions for the clinical treatment of HUA.

## 5. Conclusions

The results of this study showed that TCM can effectively lower SUA while reducing side effects and have a positive therapeutic impact on the treatment of HUA. A total of 100 HUA patients were selected as the research subjects and divided into groups A and group B, with 50 patients in each group. Group A was treated with oral allopurinol tablets, 100 mg, 2 times a day, and group B was treated with modified GSZD for two and four weeks, respectively. Results revealed that the level of blood uric acid in each group gradually dropped compared with those before treatment, and the uric acid level of all patients in group B was lower than that in group A (*P* < 0.05). Similarly, the vascular endothelial function indexes and inflammatory factor levels in each group are significantly improved compared with those before treatment, and the indexes in group B are better than those in group A. This confirms that the TCM GSZD can significantly improve the vascular endothelial function, inhibit the inflammatory response of the body, and reduce the level of SUA in patients with HUA. It is worthy of clinical promotion. There are also several limitations associated with the present study. First, the mechanism of action of GSZD is not completely known. Second, the clinical effect of GSZD on serum urate was not properly analyzed in individual male and female groups. Therefore, future studies will focus on further exploration of the mechanism of GSZD in reducing uric acid levels in both males and females.

The article "Clinical Effect of the Guizhi Shaoyao Zhimu Decoction in the Treatment of Hyperuricemia" was retracted in 2024. Reasons: signs of a paper mill; suspected computer-generated content; unreliable results or conclusions; concerns about the data.

## Figures and Tables

**Table 1:** Blood uric acid levels in groups A and B ($\bar{x}\pm s$, *μ*mol/L).

Item	Before treatment	Treatment 2 weeks	Treatment 4 weeks
Group B (*n* = 50)	465.61 ± 23.52	405.55 ± 23.91^∗^^#^	354.86 ± 18.48^∗&#^
Group A (*n* = 50)	469.35 ± 23.30	433.54 ± 16.91^∗^	383.26 ± 15.94^∗^

Note: compared with before treatment, ^∗^*P* < 0.05; compared with treatment 2 w, ^&^*P* < 0.05; compared with group A, ^#^*P* < 0.05.

**Table 2:** Vascular endothelial function indexes in each group ($\bar{x}\pm s$).

Item		MDA (nmol/mL)	NO (*μ*mol/L)
Group B (*n* = 50)	Before treatment	7.89 ± 1.82	37.37 ± 7.73
	After treatment	4.19 ± 1.00^∗^^#^	56.83 ± 7.74^∗^^#^
Group A (*n* = 50)	Before treatment	7.68 ± 1.92	35.70 ± 6.81
	After treatment	6.09 ± 1.41^∗^	41.66 ± 8.17^∗^

**Table 3:** Inflammatory factor levels in each group ($\bar{x}\pm s$).

Item		TNF-*α* (*μ*g/L)	IL-6 (*μ*g/L)	CRP (mg/L)
Group B (*n* = 50)	Before treatment	56.24 ± 3.09	40.61 ± 5.00	8.62 ± 1.27
	After treatment	26.10 ± 2.95^∗^^#^	21.36 ± 4.73^∗^^#^	3.55 ± 0.66^∗^^#^
Group A (*n* = 50)	Before treatment	56.34 ± 3.35	40.01 ± 6.07	8.71 ± 1.19
	After treatment	33.53 ± 3.15^∗^	26.77 ± 4.71^∗^	5.38 ± 1.06^∗^

**Table 4:** Comparison of 24 h uric acid levels in each group ($\bar{x}\pm s$, mmol).

Item	Before treatment	Treatment 2 weeks	Treatment 4 weeks
Group B (*n* = 50)	3.29 ± 0.59	3.54 ± 0.62^∗^^#^	3.63 ± 0.70^∗^^#^
Group A (*n* = 50)	3.11 ± 0.42	3.31 ± 0.44	3.25 ± 0.52

The article "Clinical Effect of the Guizhi Shaoyao Zhimu Decoction in the Treatment of Hyperuricemia" was retracted in 2024. Reasons: signs of a paper mill; suspected computer-generated content; unreliable results or conclusions; concerns about the data.

## Data Availability

The data that support the findings of this study are available from the corresponding author upon reasonable request.
